RETRACTED

# Growth Response in Oryctolagus cuniculus to Selenium Toxicity Exposure Ameliorated with Vitamin E

**DOI:** 10.1155/2022/8216685

**Published:** 2022-05-09

**Authors:** Rukhshanda Rehman, Nuzhat Sial, Amina Ismail, Shabir Hussain, Sobia Abid, Maryium Javed, Khansa Nadeem, Muhammad Ayoub

**Affiliations:** ^1^Department of Zoology, The Islamia University, Bahawalpur, Pakistan; ^2^School of Information Engineering, Zhengzhou University, China; ^3^School of Computer Science and Engineering, Central South University, Changsha, China

## Abstract

The adverse impacts of high temperature during the summer season on the rabbit industry have gained increased global attention. In this study, the comparative effects of biological (BIO) and chemical (CH) nanoselenium (nano-Se) combined with vitamin E on the growth and immune performances of rabbits were observed. A total of 200 white male rabbits of similar age (90 days) were divided into five treatment groups (T0, T1, T2, T3, and T4), 40 animals in each treatment. The rabbits in the first treatment group (T0) was fed basal diet; (T1) basal diet supplemented with 35 mg biological synthesized nanoselenium/kg diet; (T2) basal diet with 35 mg biological nanoselenium/kg diet+150 mg Vit. E/kg; (T3) basal diet+35 m chemically synthesized nanoselenium/kg diet; and (T4) basal diet+35 mg of chemical nanoselenium/kg diet+150 mg Vit. E/kg. The duration of this experiment was 63 days. The body weight of each rabbit was recorded weekly. Results revealed a significant (*P* < 0.05) increase in live body weight (LBW), total body gain (TBG), and feed conversion ratio (FCR) of rabbits treated with BIO-Se+Vit. E (T2) compared to the other groups. Selenium concentrations in the kidneys and liver were significantly higher (*P* < 0.05) in animals fed with BIO-Se+Vit. E (T2). The concentrations of serum urea, glutamyl transferase (GGT), and triglycerides (TG) were lower in untreated (T0) and treated groups (T1, T2, T3, and T4). From the results of this study, it can be concluded that biological nano-Se gave maximum improvement for the parameters under study compared to the chemically synthesized nanoselenium by playing a role in alleviating heat stress, increasing the growth performance, and enhancing the immunity of growing white male rabbits. Further addition of Vit. E is an alternative method to maximize productivity with no adverse effects during the fattening period of growing white male rabbits.

## 1. Introduction

Rabbit farming has an extraordinary capability and valuable contribution in enhancing meat production, meal safety, and national economy in growing nations [1]. Rabbit farming has less economic risk and is less expensive than poultry or cattle farming. It requires less space, which is much suitable for the welfare of the rural atmosphere of any country [2]. Rabbit breeder profitability has extended due to enhancing genetic selection and reproductive control [3]. The meat obtained from rabbits contains less sodium content [4] and cholesterol [5]. Regarding the amount of fat material, its meat is marked with decreasing fat, calories, and cholesterol amount [6, 7]. In summer, heat stress is the prominent problem rabbit producers face every year [8]. Sweat glands are not present on the skin of rabbits (except ear), due to which they are more sensitive to thermal stress [7]. With the rise of rabbit production, the need for animal supplements has become a necessary part of their daily diet [9]. Selenium in a hot summer environment is helpful in the antioxidant status and production [10]. As an important trace element for everyday physiological function in animals and human beings, selenium plays an essential function in growth, replica, antioxidative mechanism, hormone metabolism, anticarcinogenesis, and immunomodulation [11]. The lower level of selenium in the daily diet badly affects the working of the immune system [9]. The lower level of selenium and vitamin E deficiency result in severe disease, including Kashin-Beck disease, a form of osteoarthritis [12]. Supplementing selenium can recover this abnormality with vitamin E [12].

RETRACTED

The technology and nanotechnology are ancient and are used firstly in chemistry by the time for preparation of Roman's use of cement [13]. The concept of nanotechnology depends on decreasing particle length to change an element's physical and chemical nature [14, 15]. These days, nanoparticles are substantially considered in livestock and poultry due to chemical and physical residences [8]. Nanoparticle diameter is not more than 100 nm [15].

Vit. E is necessary for growth, better immunity, tissue cohesion, breeding, and sickness control and an antioxidant characteristic in all the body systems [1, 16]. Both Se and Vit. E are an essential and efficient antioxidant that help rabbits against lipid and protein oxidation of the outer surface membrane of different organs [17]. Combining Vit. E and Se at high value as required for nutritional requirements gives better immunity [18]. The green method proves more beneficial as compared to other chemical methods. Many types of protein pigments, multivitamins, algae carbohydrates, and lipids are present in plants. Green chemistry (plants) has been investigated successfully for metal NPs (nanoparticles) like Au, Ag, Se, MgO, CuO, and ZnO NP synthesis [19]. There are questions about using the chemical form of nano-Se [20]. The green synthesis is an environment friendly alternative to the basic chemical and physical methods as this technique removes the usage of toxic chemicals [21, 22]. Now, the synthesis of nanoparticles by the green method is a new approach that uses plants that have biomedical uses [20, 23]. To obtain the biocompatible effectiveness, this tactic is eco-friendly, safer, and easy [24]. Worldly different work has been done about the biomedical applications of selenium nanoparticles [25]. Recently, it is reported that the therapeutic margin of SeNPs has good medicinal properties and lowers the level of toxicity [26]. Researchers are studying the effects produced by BIO and CH nano-Se in growing rabbits [27]. In this study, the comparative effects of biological (BIO) and chemical (CH) nanoselenium (nano-Se) combined with Vit. E on the growth performance, serum biochemicals, and selenium metabolism (concentration of selenium in the kidneys, liver, and blood serum) of white male rabbits have been studied.

RETRACTED

## 2. Materials and Methods

### 2.1. Nanoparticle Synthesis

Biological selenium (BIO) and green method were used for the preparation of plant extract; the garlic gloves were purchased from the local market, washed with distilled water, and dried. Make a paste of garlic gloves in pistil and mortar, and add this paste into the distilled water. The prepared mixture is heated on 70 to 80°C heat for 2 to 3 hours. After preparation of the plant extract, stop heating and cool down at room temperature and filter the mixture solution by using the filter paper and use the extract for further analysis. For the preparation of selenium nanoparticles, sodium selenite (Na_2_SeO_3_) was used as the solvent throughout the experiment. The garlic extract was filtered using Whatman No. 1 filter paper. To synthesize selenium nanoparticles (SeNPs), 20 mL of the garlic extract was mixed with 100 mL of 40 mM sodium selenite solution and heated in a magnetic stirrer with 150 rpm at 60°C until the color changed to brick red after 2 to 3 days from pale yellow which designates the formation of colloidal SeNPs. After 24 h of incubation, the preparation was centrifuged at 10,000 rpm for 30 min, then washed three times with double-distilled water and ethanol [28]. Furthermore, it was dried into the oven at 60 to 70°C temperature. Released selenium nanoparticles ranged in size from a hundred to 550 nm, with an average size of 245 nm.

Chemical selenium (CH), a stock of aq. solution of ascorbic acid 50 mM, and sodium selenite 100 mM were prepared. Different ratios of ascorbic acid and sodium selenite 100 mM were combined from stock solution (1 : 1 to 1 : 6). Ascorbic acid was added to the sodium selenite solution under constant magnetic stirring at room temperature at different RPMs (200, 600, and 1000 rpm). The mixture was allowed to react in concentrated form until the colour of the solution started to change from colourless to orange. When colour was changed, the mixture was diluted by double-distilled water [24]. Analytical tools analysed the prepared particles by Raman spectroscopy UV-VIS spectroscopy.

RETRACTED

### 2.2. Animals and Experimental Groups

A total of 200 male rabbits (966 ± 12 g average body weight and 90 days old) were divided into five treatment groups (T0, T1, T2, T3, and T4), 40 animals in each treatment, each with four replicates (ten rabbits each); during the whole experimental period, hygienic environment was provided to avoid any chemical and biological infections. The first group (T0) was fed ad libitum, served as untreated (control), while in the other groups, (T1) second group diet was provided basal diet+(BIO 35 mg) biological nanoselenium/kg diet; (T2) third group diet was basal diet+(BIO 35 mg) biological nanoselenium/kg diet+50 mg Vit. E/kg; (T3) basal diet+(CH 35 mg) chemical nanoselenium/kg diet; and (T4) basal diet+(CH 35 mg) chemical nanoselenium/kg diet+150 mg Vit. E/kg. An equal amount of BIO-Se and CH-Se was used to check which method gave better effect on rabbits. Basal diet's chemical analysis was done before the beginning of the experiment. The total ingredients and the chemical composition of the basal diets are shown in Tables 1 and 2. The rabbits' diet was prepared according to requirements for the growing animals as described by the National Research Council (NRC) [29]. All the experimental animals were kept hygienic to ensure good health and avoid any parasite attack. The average ambient temperatures ranged between 30.6 and 36.0°C during the summer season, and relative humidity ranged from 68.5 to 71.0%.

### 2.3. Data Collection and Estimated Parameters

#### 2.3.1. Growth Performance

During the total experimental period, the measurements of growth performance traits were taken every week, which includes the live body weight of the rabbits (LBW), total body weight gain (TBWG), amount of feed taken by rabbits (FI), and also their feed conversion ratio (FCR).

#### 2.3.2. Economic Efficiency of the Experimental Diets

Economic efficiency can be measured according to the feed intake and the price of one kg weight. Raya equation was used to calculate the economic efficiency [15].

(1) $$\begin{array}{c} \frac{\text{Feed consumed }\left(\text{g}\right)\text{ during a certain period }}{\text{Body weight gained }\left(\text{g}\right)\text{ during the same period}}, \end{array}$$

where net revenue = selling price of weight gain (LE)–total feed cost. The selling price of weight gain = average weight gain (kg/head)∗price of one kg of live body weight (LE). Total feed cost = average feed consumption (kg/head) × price of one kg of feed (LE).

RETRACTED

#### 2.3.3. Chemical Analysis of Experimental Diets

The chemical composition of the experimental basal diet was determined in the Chemical Laboratory for Foods and Feedstuffs. Chemical analysis was performed according to the procedure described by International Standard Methods (ISO) as shown in Tables 1 and 2. Crude ash was according to ISO 5984:2002; moisture content was according to ISO 6496:1999; crude fat was according to the method described in Official Journal of the European Union (EN), 2009; crude protein was according to ISO 5983-1:2002; and crude fibre was according to the Official Journal of the European Union (EN), 2009 described method.

#### 2.3.4. Serum Biochemical, Antioxidant, and Inflammatory Indices

Blood was collected in the sterile test tubes. After the coagulation of the samples at room temperature, for about twenty minutes, centrifugation was done. After that, it was preserved. The spectrophotometric technique with diagnostic kits was used to check the serum content of different parameters under study. The determination of malondialdehyde (MDA) level of lipid peroxidation was evaluated [31].

#### 2.3.5. Sample Collection for Selenium Metabolism in Blood Serum, Kidney, Liver, and Muscles

Rabbits were selected randomly from the experimental groups to determine selenium concentration in the blood serum, kidneys, liver, and muscles. Animals have fasted for 10–12 hours before the process. Islamic method was used for slaughtering. Animals were weighed before and after they got slaughtered. Blood samples were collected from each rabbit into clean and dry nonheparinised tubes. Blood samples were centrifuged at 3000 rpm for 15 min to obtain clear serum and stored at -20°C until the determination of selenium concentration serum. Rabbits were deskinned and dressed out, and the hot carcass was taken to determine selenium concentration in the muscles, liver, and kidneys. Samples of the liver, kidneys and muscles were collected (30 g of each). Each sample was kept separately in a polythene bag with an identification card showing the sample type. Samples were transported to the laboratory to determine Se concentration in the indicated organ tissues.

### 2.4. Statistical Analysis

Data on all the parameters were subjected to ANOVA using IBM SPSS statistics (version 20) to calculate the significant difference. Mean ± SE in all the groups were subjected to post hoc Tukey's test at *P* < 0.05.

RETRACTED

## 3. Results

### 3.1. UV-Visible

The absorbance peak of nano-Se is 280 nm. In general, spherical Se NPs present peaks at around 270 nm to 300 nm linked with local surface plasm on resonance that depends on their size, morphology, and agglomeration. The UV spectrum exhibited a maximum absorption peak at 229 nm, which is attributed to the transition of the atomic C-C bonds and a shoulder peak at 300 nm is due to the n-transition of the C-O group. The absorbance peak for BIO-Se and CH-Se has been shown in Figures 1 and 2.

### 3.2. Effects of Biologically and Chemically Synthesized Nanoselenium with Vit. E on Growth

The results showed that biological and chemical nanoselenium supplementation along vitamin E caused a significant increase in live body weight at weeks 14, 16, 18, and 20 of the experiment. In comparison, biologically synthesized selenium gave better results than CH-selenium on growth. The same results with the addition of Vit. E, rabbits of group T2 (BIO-selenium with Vit. E) showed a significant (*P* < 0.05) increase in growth than T4 (CH-selenium with Vit. E), as shown in Table 3.

The result shows that the total body weight gain (TBWG) of white male was significantly (*P* < 0.05) increased in the T2 group (BIO-Se with Vit. E supplementation) and T4 group (CH-selenium with Vit. E supplementation) in our experimental study as shown in Table 4.

Feed intake was significantly high in the T2 group (BIO-se with Vit. E supplemented), followed by the T4 group as shown in Table 5.

The feed conversion ratio was significantly (*P* < 0.05) improved in groups T2 (BIO-Se along with Vit. E) and T4 (CH-Se along with Vit. E), as shown in Table 6.

### 3.3. Blood Serum Metabolite

The T2 (BIO-Se with Vit. E) group has a significantly lowered (*P* < 0.01) serum urea content in comparison to the other groups (T1, T3, and T4) and T0 group. The highest values were recorded with T0 (control), while the T1 (BIO-Se), T3 (CH-selenium), and T4 (CH-Se with Vit. E) treatments gave medium values. The treatments of BIO-Se with Vit. E (T2) and CH-Se (T3) produced the reduced values of TG and GGT in the blood serum of white male rabbits. Furthermore, the highest TG and GGT were in the CH-Se with the Vit. E (T3) and control group (T0), respectively. Not any significant effect on the total bilirubin, direct and indirect bilirubin was observed in the serum of white male rabbits by any additive, as shown in Table 7.

### 3.4. Antioxidant Parameters

The level of SOD was significantly lowered by supplementation of nano-Se. The T1 (BIO-Se) and T2 (BIO-Se with Vit. E) groups gave decreased values for the level of SOD than the other groups. The antioxidant indicators' maximum values were in T0 (control group). The other white male rabbit (except T4) had significantly lowered for the production of nitric oxide (NO) and MDA as compared to T0 (control group). The CAT levels were improved in growing white male rabbits after supplementation with nano-Se (CH-Se, BIO-Se) as shown in Table 7.

RETRACTED

### 3.5. Selenium (Se) Concentration in the Kidney, Liver, Body Muscles, and Blood Serum of Rabbits

The concentration of selenium was significantly (*P* < 0.05) increased in the group of rabbits fed BIO-Se with Vit. E (T2) and T4 (CH-Se with Vit. E). Addition of Vit. E results in a higher concentration of selenium in the kidney and liver. On the other hand, in blood serum and body muscle, selenium concentration increases significantly in group T1 (BIO-selenium) and T3 (CH-Se), as shown in Table 8.

### 3.6. Economic Efficiency of the Experimental Diets

The obtained results showed that BIO-Se supplementation was beneficial in achieving the highest economic efficiency and the groups having BIO-selenium with Vit. E and CH-Se with Vit. E fed gave the lowest economic efficiency. Addition of Vit. E decreased economic efficiency as shown in Table 9.

The selling price of live body weight for rabbits = 40 LE/kg; price of the diet without additive = 4.2 LE/kg; price of the diet with Vit.E = 4.35 LE/kg; price of the diet with chemical nanoselenium = 4.23 LE/kg; price of diet with chemical nanoselenium and Vit.E = 4.55 LE/kg; price of diet with biological nanoselenium = 4.32 LE/kg; and price of the diet with biological nano − selenium&Vit.E = 4.65 LE/kg.

## 4. Discussion

The rabbit industry has suffered a lot due to global warming; their economic profit and productivity get disturbed [32]. Different dietary manipulations are used to overcome the negative influences of heat stress in rabbits [33]. In animals with a lower Se level suffering from different diseases, GSH Px activity in organs and tissues decreased [12].

There are different methods for the synthesis of nano-Se. Chemically synthesized nano-Se has been widely used in animals. The conventional methods used to produce NPs are toxic, expensive, and nonenvironment friendly. To overcome these problems, researchers have found the green routes, i.e., the naturally occurring sources and their products that can be used to synthesize NPs [34].

The present research shows that feeding biological nano-Se helped to improve LBW, BWG, and FCR in heat-stressed rabbits compared to the chemical nano-Se and control. However, this study agrees with the result stated by Sheiha et al. who reported that improved effects showed for biologically synthesized selenium as compared to the chemically synthesized and reported BIO-selenium (25 or 50 mg/kg) have better growth and LBW as compared to the CH-selenium (25 or 50 mg/kg) and control groups of growing rabbits [27].

RETRACTED

Several studies support that addition of nano-Se separately as well as in combination with other dietary manipulations results in the enhanced growth of the rabbits. The addition of selenium to the diet of the rabbits results in enhanced FCR and reduced FI [18]. In a study, it is stated that the addition of 0.70 mg/kg selenium to the diet of the rabbits results in enhanced growth parameters [24]. The authors in [3] reported that the combination of nanoselenium with prevalent garlic oil and much better results were obtained in the BW bodyweight of rabbits [32]. In another study, it is stated that the combination of nanozinc and nanoselenium gave better results in the growth of the rabbits as compared to the control group [9] and reported that diet with 60 mg nanozinc or 0.3 mg nanoselenium had a maximum value of growth parameters. In a study, it is reported that a combination of organic and inorganic selenium had higher live body weight (LBW) growth (*P* < 0.05), good feed conversation ratio (FCR), and total body weight gain (TBWG) [10]. Elkholy et al. studied the comparison of different forms of selenium used as a supplement in the diet of rabbits and their overall effect on production, and they concluded that selenium in either form organic or inorganic form put beneficial effects on survival, on growth rate, and in the meat of rabbits [4]. Addition of Vit. E in this study showed a significant (*P* < 0.05) increase in growth. It is stated that the addition of Vit. E results in increased body weight [35, 36], and that agrees with the results. Dalle Zotte and Szendrő interpreted the improvement in body weight by dietary addition of Vit. E [37]. Rooke et al. and Ebeid et al. studied that Vit. E is essential for growth, immunity characteristic increase, tissue cohesion, breeding, sickness control, and having an antioxidant characteristic in all the body systems [1, 16]. Marounek et al. and Ebeid et al. reported that live body weight and total weight gain have remarkable effects by adding the Vit. E [1, 38]. Shara et al. worked on the effect of selenium plus Vit. E along with AD3E vitamins and concluded that diet supplemented with Vit. E improved BW (*P* < 0.005) and decreased (*P* < 0.001) daily water intake [39].

The administration of nano-Se (BIO-selenium with Vit. E or CH-selenium) reduced the level of blood urea as compared to the T0 group, results of GGT and TG for rabbits fed (BIO-selenium, BIO-selenium with Vit. E, or CH-selenium) were decreased than the T0 group. Concerning the liver and kidney functions, level of creatinine and total, indirect ,and direct bilirubin did not show any remarkable changes. Abdel-Wareth et al. reported that the group of rabbits fed with nanoselenium had a lower level of urea [32]. Additionally, a significant reduction was reported in the TG level as a response to nano-Se supplementation in broiler chicks [40]. Our results concluded that nano-Se improved liver and kidney functions, thus alleviating the adverse influences of a hot environment.

RETRACTED

In conclusion, the dietary addition of nanoselenium led to increased concentrations of total protein in the blood serum of white male rabbits. This result aggress with the work of [41]. It was reported that supplementation of nanoselenium increases the amount of total protein in the blood [42]. This result disagrees with the work of Šperanda et al. They reported that there is no significant change or increase in the total protein level of blood by supplementation of nanoselenium [43].

In our study, feeding rabbits with nanoselenium improved the antioxidant activities by significantly increasing the activities of GSH and CAT in comparison to the heat stress group and also decreased the level of NO and MDA in the groups (BIO-selenium, BIO-selenium with Vit. E, or CH-selenium) as compared to the other groups. El-Deep et al. [44] reported that fed nano-Se (0.2–0.3 mg/kg) in poultry improved the reduced glutathione (GSH-P) activity in the blood serum. Zhou et al. stated that Se supplementation contributes to several immune functions, such as reducing the levels and duration of inflammatory infections, minimising glucocorticoids (which are an indicator for immunity disorder) [45] and also the arrangement of the function of T lymphocyte cells. Se is an essential trace element for combating oxidative stress, hence the cell's redox state, due to its integration as selenocysteine into GSH-Px [46].

Our results showed that biological nano-Se and Vit. E increase selenium concentration in the kidney and liver. In contrast, Se concentration in muscles and blood serum was not significantly affected by Vit. E addition to the diet. The result agrees with the previous work of Abd Allah et al. who reported that adding Vit. E to the basal diet significantly (*P* < 0.05) increased level of Se in the kidneys and liver of all rabbit groups.

The result disagreed with the previous research of Ebeid et al. and ElKholy et al., who observed that the concentration of Se (g/kg) in the hind leg significantly increased (*P* < 0.05) in rabbits fed the diet supplemented with selenium plus Vit. E compared with those fed with diet Vit. E only [1, 4].

Abdel-Wareth et al. reported that basal diet fed with selenium and garlic oil to the growing rabbits results in improved and efficient kidney and liver functions [32]. Sheiha et al. concluded that supplementation of nanoselenium improves liver and kidney functions and decreases the adverse effect of hot temperature [27].

RETRACTED

Abdel-Wareth et al. reported that being fed with nanoselenium results in a lower level of urea in the kidneys and liver than the control [32]. Lee et al. stated that GSH-Px non-selenium-dependent forms are more present in the liver and kidney of rabbits [47]. On the other side, the lungs, heart, and blood serum have only selenium-dependent GSH-Px activity.

El-Deep et al. and Lebas et al. reported that reducing the oxidative pressure on different organs of rabbits is more relayed on Vit. E and significantly less on selenium [48]. Abd Allah et al. stated that basically, selenium moves from the blood into tissues and presents in protein in the kidney, liver, muscles, and blood serum [49].

Economic efficiency was highest in BIO-selenium supplemented groups and lowest in Vit. E supplemented groups. It is reported that the highest economic efficiency was recorded with rabbits fed supplemental nanoselenium [50]. Abd Allah et al. reported that economic efficiency was lowest for the rabbits fed Org-Se plus Vit. E compared to the other groups [49].

El-Monie et al. reported that the economic feed efficiency in their study showed that using BET, VC, or VE in the growing rabbit diets was more economical than the nonsupplemented diets [41]. Ebeid et al. indicated that EE was highest for rabbits fed with the nanoselenium compared to the other group fed with organic selenium and the control group [1]. Abd Allah et al. reported that from the economic point of view to ameliorating the adverse effects of heat stress on growing rabbits during the hot summer conditions in Egypt, it is advisable to supply the basal rabbit diet with Se, either as nano-Se or Org-Se only without Vit. E diet [49].

## 5. Conclusion

In view of the above findings, nano-Se is an essential element that helps growing white male rabbits to cope with heat stress's adverse effects. The best results in this study were retrieved for BIO-Se compared to the CH-Se. Growth parameters increased significantly with BIO-selenium with Vit. E, T2 group. So in the light of this study, we conclude that supplementation of BIO-Se with Vit. E improves growth and antioxidant status and regulates the inflammatory cytokine responses and selenium metabolism in growing white male rabbits. Moreover, the addition of Vit. E also plays an important antioxidant role along with selenium.

## Figures and Tables

**Figure 1:** UV-visible spectrum of Se NPs (green synthesis).

RETRACTED

**Figure 2:** UV-visible spectrum of Se NPs (chemical synthesis).

**Table 1:** Chemical composition of the basal experimental diet.

Items (ingredients)	Content (%)
Clover hay	39.50
Bone meal	0.75
Wheat bran	30.00
Calcium carbonate	0.68
Yellow corn	12.00
Sodium chloride	0.57
Soybean meal (44%)	12.00
Vitamins and mineral	0.34
Molasses	4.00
1 DL-methionine	0.16
Total	100

**Table 2:** Chemical composition of the basal experimental diet.

Items (ingredients)	Chemical composition (%)
Dry matter (DM)	90.23
Crude protein (CP)	17.07
G.E (kcal/kg)^∗∗^	2600
Crude fibre (CF)	15.25
Ether extract (EE)	3.03
Nitrogen-free extract (NFE)	50.51
Total phosphorous (P)	0.50
Total calcium (a)	0.90
Ash	7.45
Methionine+cysteine^∗∗∗^	0.66
Lysine^∗∗∗^	0.90

^∗^Each 3 kilograms of premix contains Vit. A 12000000 IU, Vit. D 31500000 IU, Vit. E 50 g,Vit. K 32 g,Vit. B1 2 g, Vit. B2 6 g, Vit. B12 0.01 g, Chol. Chlod 1200 g, biotin 0.2 g, niacin 50 g, pantothenic acid 20 g, folic acid 5 g, magnesium 400 g, Copper 5 g, iodin 0.75 g, selenium 0.2 g, iron 75 g, manganese 30 g, and zinc 70 g. ^∗∗∗^It was determined according to [30]. ^∗∗∗∗^It was calculated according to [29].

**Table 3:** Effect of biological and chemically synthesized nanoselenium with Vit. E on live body weight (LBW; g) of the growing rabbits at different ages (mean ± SE).

Weeks	T0 (control)	T1	T2	T3	T4
12	958.22 ± 3.61	972.43 ± 4.52	1002.82 ± 4.07^∗^	960.01 ± 6.17	996.03 ± 2.21^∗^
14	1224.24 ± 4.65	1236.09 ± 5.02	1288.43 ± 7.68^∗^	1240.32 ± 7.16	1271.98 ± 7.40^∗^
16	1511.09 ± 4.63	1538.98 ± 4.29	1594.65 ± 5.55^∗^	1518.19 ± 6.83	1573.03 ± 6.78^∗^
18	1880.08 ± 6.43	1895.01 ± 5.37	1995.23 ± 6.78^∗^	1904.95 ± 4.28	2158.92 ± 7.02^∗^
20	2106.98 ± 6.25	2111.65 ± 3.97	2171.04 ± 6.00^∗^	2121.03 ± 6.64	2142.09 ± 6.37^∗^

**Table 4:** Effect of biologically and chemically synthesized nanoselenium with Vit. E on total body weight gain (TBWG; g) of the growing rabbits at different ages (mean ± SE).

Weeks	T0 (control)	T1	T2	T3	T4
12–14	26.11 ± 5.75	27.51 ± 6.09	36.53 ± 11.80^∗^	30.54 ± 8.80	34.33 ± 10.09^∗^
15–16	28.21 ± 5.41	28.34 ± 5.67	31.26 ± 9.84^∗^	29.20 ± 11.68	33.43 ± 10.64^∗^
17–18	26.04 ± 8.88	27.71 ± 4.96	32.56 ± 7.38^∗^	28.06 ± 7.18	30.41 ± 9.36^∗^
19–20	24.84 ± 7.99	26.91 ± 5.99	35.05 ± 7.22^∗^	28.75 ± 8.27	32.16 ± 11.18^∗^

**Table 5:** Effect of biologically and chemically synthesized nanoselenium with Vit. E on feed intake (FI; g) of the growing rabbits at different ages (mean ± SE).

Weeks	T0 (control)	T1	T2	T3	T4
12–14	78.9 ± 3.05	80.09 ± 2.06	90.03 ± 2.83^∗^	78.09 ± 1.87	99.91 ± 1.74^∗^
15–16	84.07 ± 1.45	81.71 ± 1.65	92.70 ± 1.48^∗^	86.17 ± 1.79	98.49 ± 2.28^∗^
17–18	98.51 ± 2.80	96.19 ± 1.90	122.84 ± 2.56^∗^	98.19 ± 2.27	105.04 ± 1.68^∗^
19–20	85.11 ± 2.04	83.61 ± 1.76	118.03 ± 1.65^∗^	87.61 ± 1.82	109.48 ± 1.48^∗^

RETRACTED

**Table 6:** Effect of biologically and chemically synthesized nanoselenium with Vit. E on feed conversion ratio (FCR; g feed/g gain) of the growing rabbits at different ages (mean ± SE).

Weeks	T0 (control)	T1	T2	T3	T4
12–14	4.1 ± 0.17	3.18 ± 0.10	5.15 ± 0.16^∗^	3.75 ± 0.13	5.81 ± 0.15^∗^
15–16	4.09 ± 0.10	3.11 ± 0.09	5.0 ± 0.09^∗^	3.9 ± 0.24	5.02 ± 0.24^∗^
17–18	4.09 ± 0.11	3.84 ± 0.122	5.41 ± 0.12^∗^	3.83 ± 0.13	5.05 ± 0.13^∗^
19–20	4.16 ± 0.15	3.58 ± 0.11	5.55 ± 0.13^∗^	3.58 ± 0.12	5.09 ± 0.19^∗^

**Table 7:** Effect of biologically and chemically synthesized nanoselenium with Vit. E on blood serum metabolites (mean ± SE).

Items	T0 (control)	T1	T2	T3	T4
Creatinine (mg/dL)	1.45 ± 0.21	4.14 ± 0.33^∗^	1.12 ± 0.24	1.25 ± 0.20	2.34 ± 0.19^∗^
Urea (mg/dL)	52.8 ± 0.06	51.1 ± 0.11	44.84 ± 0.12^∗^	49.41 ± 0.09	51.33 ± 0.14
GGT (U/L)	5.36 ± 0.03	5.01 ± 0.09	4.73 ± 0.12^∗^	4.94 ± 0.03	5.47 ± 0.06
TG (mg/dL	144 ± 0.21	75.43 ± 0.17^∗^	73.08 ± 0.11^∗^	73.73 ± 0.09^∗^	107.32 ± 0.08^∗^
Total protein (mg/dL)	4.08 ± 0.21	5.86 ± 0.27^∗^	5.44 ± 0.31^∗^	5.79 ± 0.24^∗^	5.66 ± 0.33^∗^
Albumin (mg/dL)	2.11 ± 0.10	3.55 ± 0.11^∗^	3.14 ± 0.09^∗^	3.41 ± 0.11^∗^	3.34 ± 0.11^∗^
Globulin (mg/dL)	1.87 ± 0.07	2.33 ± 0.06^∗^	2.3 ± 0.09^∗^	2.42 ± 0.08^∗^	2.31 ± 0.06^∗^
Total bilirubin (mg/dL)	0.87 ± 0.11	0.88 ± 0.06	0.810.09	0.83 ± 0.06	0.89 ± 0.77
Direct bilirubin (mg/dL)	0.2 ± 0.01	0.19 ± 0.04	0.21 ± 0.07	0.21 ± 0.08	0.2 ± 0.03
Indirect bilirubin (mg/dL)	0.75 ± 0.03	0.76 ± 0.09	0.73 ± 0.11	0.73 ± 0.07	0.7 ± 0.13
NO (*μ*mol/L)	0.25 ± 0.05	0.19 ± 0.07^∗^	0.19 ± 0.04^∗^	0.21 ± 0.04	0.23 ± 0.09
MDA (nmol/mL)	0.3 ± 0.02	0.25 ± 0.11^∗^	0.23 ± 0.09^∗^	0.21 ± 0.07^∗^	0.28 ± 0.12^∗^
SOD (U/mL)	0.28 ± 0.03	0.23 ± 0.05^∗^	0.21 ± 0.08^∗^	0.24 ± 0.06	0.26 ± 0.04
GSH (ng/mL)	0.12 ± 0.06	0.15 ± 0.02^∗^	0.15 ± 0.10^∗^	0.18 ± 0.16^∗^	0.11 ± 0.13
CAT (ng/mL)	0.2 ± 0.08	0.15 ± 0.06	0.24 ± 0.02	0.28 ± 0.01	0.05 ± 0.07^∗^

^∗^NO: nitric oxide; MDA: malondialdehyde; GSH: reduced glutathione; SOD: superoxide dismutase; CAT: catalase.

**Table 8:** Concentration (*μ*g/kg) of selenium in the liver, kidney, and blood serum of the growing rabbits at different ages (mean ± SE).

Items	T0 (control)	T1	T2	T3	T4
Kidneys	3.98 ± 1.6	4.64 ± 2.1	8.09 ± 2.0^∗^	4.61 ± 1.5	7.24 ± 0.9^∗^
Liver	3.42 ± 0.6	4.41 ± 1.5	7.89 ± 1.9^∗^	4.9 ± 0.24	6.08 ± 1.2^∗^
Muscles	2.4 ± 0.9	4.12 ± 1.7^∗^	3.08 ± 0.7	4.42 ± 0.6^∗^	3.32 ± 1.3
Blood serum	3.36 ± 0.7	5.84 ± 0.8^∗^	4.41 ± 1.6	5.91 ± 0.9^∗^	4.07 ± 0.7

**Table 9:** Effect of biologically and chemically synthesized nanoselenium with Vit. E on economic efficiency (EE) at different ages of growing rabbits.

Weeks	T0	T1	T2	T3	T4
12–14	210	280	198	244	184
15–16	324	377	284	339	268
17–18	160	245	148	210	133
19–20	282	349	242	311	227

RETRACTED

## Data Availability

Data is openly available for readers.
